The article "Effect of Conventional Nursing Combined with Bedtime Oculomotor Training on Sleep Quality and Body Immunity of Advanced Lung Cancer Patients" was published in 2022. Journal: J Healthc Eng.

# Effect of Conventional Nursing Combined with Bedtime Oculomotor Training on Sleep Quality and Body Immunity of Advanced Lung Cancer Patients

**DOI:** 10.1155/2022/4357915

**Published:** 2022-03-10

**Authors:** Haiping Hu, Xing Zhang, Ling Chen, Rongfeng Liu, Ting Liu, Shuai Li, Huixia Xu

**Affiliations:** ^1^Department of Oncology, The Fourth Hospital of Hebei Medical University, Shijiazhuang 050011, Hebei, China; ^2^Department of Cancer Center, Union Hospital, Tongji Medical College, Huazhong University of Science and Technology, Wuhan 430000, Hubei, China; ^3^Department of Nursing, The Fourth Hospital of Hebei Medical University, Shijiazhuang 050011, Hebei, China

## Abstract

**Objective:**

The aim of this study is to explore the effect of conventional nursing combined with bedtime oculomotor training on sleep quality and body immune of advanced lung cancer patients.

**Methods:**

By means of a retrospective study, 120 advanced lung cancer patients admitted to our hospital from January 2019 to January 2020 were selected as the research subject and divided into the intervention group (PSQI (Pittsburgh Sleep Quality Index) score≥10 points, *n* = 60) and the control group (PSQI score<10 points, *n* = 60). Conventional nursing was performed to the control group, and an eye movement exercise before sleep was added additionally in the intervention group, 30 min each time, once a day, and 5 times a week for 3 months, so as to compare their sleep quality, body immunity indexes, negative emotion scores, adverse reaction rate (ARR), quality of life, and satisfaction with nursing.

**Results:**

After nursing, the intervention group obtained a significantly lower PSQI score (5.54 ± 1.23 VS 7.98 ± 1.65, *P* < 0.05), better body immunity indexes (*P* < 0.001), lower negative emotion scores (*P* < 0.05), lower ARR (*P* < 0.05), better quality of life (*P* < 0.001), and higher satisfaction with nursing (*P* < 0.05) than the control group.

**Conclusion:**

Combining conventional nursing with the eye movement exercise before sleep can alleviate negative emotions, improve the sleep quality, promote body immunity, and reduce the ARR, which is more satisfying to patients and should be applied and promoted in practice.

## 1. Introduction

Lung cancer is a relatively common malignancy in clinical practice, and the number of patients who develop lung cancer has been increasing worldwide in recent years, with Chinese lung cancer patients accounting for approximately 1/3 of them, indicating that this disease has become a serious problem in social medical care in China, threatening the physical health of Chinese residents [1–3]. After lung cancer developed into the advanced stages, chemotherapy has become the main treatment modality for patients, which can relieve the clinical symptoms of patients and prolong their survival, but long-term chemotherapy will reduce their body's immunity and lead to all types of toxic side effects, seriously affecting the physical and mental status of patients. Besides, Gentry *M* T and other scholars found that long-term illness also causes patients to develop a bipolar mood [4], which combined with various factors such as cancer fatigue is highly likely to cause sleep disturbance in patients with advanced lung cancer, whose quality of survival will be further reduced. Therefore, there is a great need for intervening scientific and efficient nursing measures to reduce the physical and mental burden on patients [5, 6]. Conventional chemotherapy care is dominated by the completion of treatment tasks and does not make individual interventions on patients' sleep disturbance, so little improvement has been observed in the sleep of advanced lung cancer patients, while studies of some scholars in recent years have reported that oculomotor training can improve patients' brain oxygen supply and enhance their self-efficacy [7, 8]. The oculomotor training refers to the scientific and regular eye movement training, which is able to improve ocular blood circulation and is often used in patients with ocular neuropathy and sleep disorders. Studies have shown that oculomotor training can improve the quality of sleep in diabetic patients [9, 10]. Based on this, to explore the effect of conventional nursing combined with bedtime oculomotor training on sleep quality and body immunity of advanced lung cancer patients, 120 advanced lung cancer patients admitted to our hospital from January 2019 to January 2020 were selected for the study, with the results summarized as follows.

## 2. Materials and Methods

### 2.1. General Information

Under the guidance of World Medical Association Declaration of Helsinki [11], 120 advanced lung cancer patients admitted to our hospital from January 2019 to January 2020 were selected and divided into the intervention group (PSQI scores≥10 points, *n* = 60) and the control group (PSQI scores<10 points, *n* = 60), with no statistical differences in their general information (*P* > 0.05); see Table 1. The study was approved by the Hospital Ethics Committee.

### 2.2. Inclusion Criteria

The inclusion criteria of the study were as follows. (1) fully understood the study process and signed the informed consent; (2) diagnosed with the advanced lung cancer and accepted chemotherapy in our hospital [12]; and (3) the estimated survival was at least 3 months [13].

### 2.3. Exclusion Criteria

The exclusion criteria for the patients in the study were as follows. (1) presence of mental problems or inability to communicate with others; (2) suffering from other organic diseases; (3) presence of coagulation disorders [14]; (4) presence of immune system abnormalities; and (3) presence of other failures to cooperate with the study [15].

### 2.4. Methods

Conventional nursing was performed in the control group for three months with the following steps. (1) Reading the patients' personal information repeatedly to grasp their conditions and establish nursing measures with a personalized difference. (2) Introducing chemotherapy to patients according to their degree of awareness to clear their confusion and enhance their initiative in treatment. (3) Paying close attention to patients' psychological state and listening to their subjective demand to timely resolve their depression and intervene in psychological treatment immediately in case of presenting severe psychological problems. (4) Conducting medication intervention to patients as directed to guide the patients to follow the correct dietary plan and exercise plan, and carrying out health education to the patients and their family members to improve the quality of home care.

Three-month bedtime oculomotor training was added in the intervention group additionally with the following steps. (1) Nursing personnel should give oculomotor training promotion and education to patients, so that patients could understand the importance of oculomotor training and enhance their training cooperation. (2) Nursing personnel should guide the patients to do the oculomotor training, namely, to move their eyeballs inward, inward + upward, inward + downward, outward + upward, and outward + downward before sleep for 30 minutes each time, once a day and 5 times a week. (3) Nursing personnel should establish a sleep index sheet at the foot of the bed for dynamic observation; daily evaluation was conducted 24 hours before chemotherapy and during chemotherapy, and discharge evaluation and guidance were conducted before discharge.

### 2.5. Observation Criteria

1. Sleep quality. Before and after nursing, patients' sleep was evaluated by PSQI (Pittsburgh Sleep Quality Index), covering 7 dimensions including sleep quality, bed time, hours of sleep, and daily mental state. On a scale of 0–21 points, higher scores indicated a worse sleep condition [16].
2. Body immunity indexes. T lymphocyte subsets CD3^+^, CD4^+^, CD4^+^/CD8^+^ levels in patients of both groups were compared before and after nursing [17].
3. Negative emotion scores. Before and after nursing, the patients' negative emotions were evaluated with the Self-Rating Anxiety Scale (SAS) and Self-Rating Depression Scale (SDS), each contained 20 items and had a total score of 100 points, with higher scores indicating more serious negative emotions [18].
4. Adverse reaction rate (ARR). The adverse reactions included nausea and vomiting, poor appetite, diarrhea, granulocytopenia, and stomatitis, and the numbers of patients with adverse reactions were counted.
5. Quality of life. The Generic Quality of Life Inventory-74 (GQOI-74) was adopted as the scoring basis, which covered the social function, physical function, psychological function, and material life, and each dimension was rated on a 100-point scale, with higher scores indicating a better quality of life [19].
6. Patient satisfaction with the nursing. Nursing quality, manners, and service contents were assessed using the scale proposed by our hospital. Ranging from 0 to 5 stars, 5 stars denoted fully satisfied, 3–4 stars denoted satisfied, and 2 stars and less denoted dissatisfied. The number of satisfied patients was counted.

### 2.6. Statistical Processing

In this study, the data processing software was SPSS20.0, the picture drawing software was GraphPad Prism 7 (GraphPad Software, San Diego, USA), items included were enumeration data and measurement data, methods used were X^2^ test and *t*-test, and differences were considered statistically significant at *P* < 0.05.

## 3. Results

### 3.1. Comparison of Patients' Sleep Quality

After nursing, the sleep quality of the intervention group was significantly better than that of the control group (*P* < 0.001); see Figure 1.

In Figure 1, the horizontal axis from left to right indicated before and after nursing, and the vertical axis indicated the PSQI score (points); the lines with dots indicated the intervention group, and the lines with blocks indicated the control group; and ∗ indicated *P* < 0.001.

Before nursing, the PSQI scores of both groups were not statistically different (10.23 ± 2.54 vs 10.65 ± 2.50, *P* > 0.05), and after nursing, the PSQI scores of the intervention group were significantly lower than those of the control group (5.54 ± 1.23 vs 7.98 ± 1.65, *P* < 0.05).

### 3.2. Comparison of Patients' Body Immunity Indexes

After nursing, the body immunity indexes of the intervention group were significantly better than those of the control group (*P* < 0.001); see Table 2.

### 3.3. Comparison of Patients' Negative Emotion Scores

After nursing, the negative emotion scores of the intervention group were significantly lower than those of the control group (*P* < 0.05), see Table 3.

### 3.4. Comparison of Patients' ARR

The ARR of the intervention group was significantly lower than that of the control group (*P* < 0.05); see Figure 2.

In Figure 2, the black areas indicated nausea and vomiting, the dark gray areas indicated poor appetite, the light gray areas indicated diarrhea, the white areas indicated granulocytopenia, and the grid areas indicated stomatitis; the left figure indicated the intervention group, and the right figure indicated the control group.

The number of patients with nausea and vomiting in the intervention group was significantly lower than that in the control group (18 (30.0%) vs 30 (50.0%), *P* < 0.05);

The number of patients with a poor appetite in the intervention group was significantly lower than that in the control group (20 (33.3%) vs 32 (53.3%), *P* < 0.05);

The number of patients with diarrhea in the intervention group was significantly lower than that in the control group (5 (8.3%) vs 20 (33.3%), *P* < 0.05);

The number of patients with granulocytopenia in the intervention group was significantly lower than that in the control group (17 (28.3%) vs 28 (46.7%), *P* < 0.05).

The number of patients with stomatitis in the intervention group was significantly lower than that in the control group (20 (33.3%) vs 35 (58.3%), *P* < 0.05).

### 3.5. Comparison of Patients' Quality of Life

After nursing, the quality of life of the intervention group was significantly better than that of the control group (*P* < 0.001); see Figure 3.

In Figure 3, the horizontal axis from left to right indicated before and after nursing, and the vertical axis indicated the GQOI-74 score (points); the black areas indicated the intervention group, and the gray areas indicated the control group; and ^*∗*^indicated *P* < 0.001.

Before nursing, the GQOI-74 scores of both groups were not statistically different (62.65 ± 5.54 vs 61.98 ± 5.65, *P* > 0.05), and after nursing, the GQOI-74 scores of the intervention group were significantly lower than those of the control group (95.65 ± 2.54 vs 81.55 ± 4.98, *P* < 0.001).

### 3.6. Comparison of Patient Satisfaction with Nursing

The patient satisfaction with nursing of the intervention group was significantly higher than that of the control group (*P* < 0.05); see Table 4.

## 4. Discussion

Lung cancer can be caused by many factors. With the continuous change of the world environment in recent years, the number of patients suffering from lung cancer is increasing progressively year by year, and the disease has now become the one affecting life and health the most [20]. Chemotherapy is an important way to improve the condition of late lung cancer patients and is the first choice to prolong their survival, but long-term chemotherapy can lead to nausea, vomiting, and other body reactions as well as aggravated adverse emotions, significantly affecting their quality of life in a negative way [20–22]. Increased research into approaches to the care of these patients is important as studies have demonstrated that more than 50% of them tend to have sleep disturbance, and the odds may even be increased if they accept chemotherapy in hospital accompanied by an aggravated mental burden [23].

The care of patients with advanced cancer mostly aims at the completion of treatment, and nowadays, with the advancement of humanities, psychological nursing is becoming more popular in the clinic. Psychological nursing can improve the negative emotions of advanced cancer patients to a certain extent, so that the patients' depression can be released, explaining the fact that the psychological state after nursing was improved in both groups. Moreover, in the intervention group, it was even better because bedtime oculomotor training could help the patients concentrate, improve their self-efficacy through aerobic exercise of the brain, and re-establish a peace mind in an easy and quiet training environment. Because negative emotions are an important factor affecting the quality of sleep in advanced lung cancer patients, when patients become less anxious, their time taken to fall asleep is also reduced, thereby lifting the quality of sleep. Moreover, bedtime oculomotor training can increase eye fatigue and elevate the ocular blood circulation level, making it less difficult for the patients to fall asleep; hence, the quality of sleep after nursing in the intervention group was significantly better than that in the control group (*P* < 0.001).

There is a close relationship between sleep quality and treatment effect in advanced lung cancer patients, and many studies have confirmed that sleep quality is a critical indicator affecting patient outcomes. Palesh Oxana et al. found that sleep quality was generally lower in patients who had undergone cancer surgery, and intervention measures could enhance sleep quality in cancer patients who received chemotherapy [24]. A good sleep elevates the patients' body tolerance and refreshes them with a better mental state during daytime, whereas poor sleep results in a disturbed biological clock and more fatigue. In this study, the results showed that the sleep quality and body immunity of the intervention group after nursing were significantly better than those of the control group (*P* < 0.001), indicating that with better body recovery and lowered body energy consumption, the tolerance to chemotherapy of patients could be improved obviously.

The study also concluded that the quality of life of the intervention group after nursing was significantly better than that of the control group (*P* < 0.001), which was consistent with the founding of Bowden *J* et al. In their study, the patients in the experimental group accepted conventional nursing combined with oculomotor training, and the patients in the control group accepted conventional nursing only, and the results showed that the quality of life after nursing of the experimental group was obviously higher than that of the control group (95.87 ± 2.11 vs 80.57 ± 4.12, *P* < 0.001) [25], indicating that the combined mode could promote the quality of life and patient satisfaction with nursing by improving their sleep quality and enhancing their body immunity. Widely applying the conventional nursing combined with oculomotor training can lower the possibility of nursing disputes and provide patients with more efficient and scientific nursing.

In conclusion, sleep quality occupies an important position in the treatment of cancer patients and is closely related to the prognosis of patients. Conventional nursing combined with bedtime oculomotor training can alleviate the negative emotions of advanced lung cancer patients, improve their sleep quality, and promote their body immunity, thereby lowering the adverse reaction rate and lift patient satisfaction with the nursing, which should be promoted and applied in practice.

## Figures and Tables

**Figure 1:** Comparison of patients' sleep quality ($\bar{\text{x}}$ ±*s*, points).

**Figure 2:** Comparison of patients' ARR.

**Figure 3:** Comparison of patients' quality of life ($\bar{\text{x}}$ ±*s*, points).

**Table 1:** Comparison of patients' general information.

Group	Intervention group (*n* = 60)	Control group (*n* = 60)	X^2^/*t*	*P*
*Gender*				
Male	32	33	0.034	0.855
Female	28	27		

Mean age (years old)	50.12 ± 5.68	51.62 ± 5.64	1.452	0.149
Mean duration of disease (years)	2.98 ± 2.10	3.10 ± 2.11	0.312	0.755

*TNM stage*				
IIIb	35	34	0.034	0.853
IV	25	26		

*Tumor type*				
Squamous cell carcinoma	25	26	0.034	0.853
Small cell carcinoma	13	13	<0.001	1.000
Adenocarcinoma	22	21	0.036	0.849

*Basic disease*				
Diabetes	10	9	0.063	0.803
Coronary heart disease	8	9	0.069	0.793
Hypertension	14	13	0.048	0.827
Others	10	11	0.058	0.810

*Educational degree*				
Junior high school and below	15	14	0.046	0.831
Senior high school	25	26	0.034	0.853
College and above	20	20	<0.001	1.000

*Monthly income (yuan)*				
≥3000	24	25	0.035	0.853
<3000	36	35		

**Table 2:** Comparison of patients' body immunity indexes ($\bar{\text{x}}$ ±*s*).

Category	Intervention group		Control group		t	*P*
CD3^+^ (%)	Before	60.11 ± 2.21	Before	59.68 ± 2.35	1.032	0.304
	After	43.25 ± 2.65	After	50.65 ± 2.65	15.295	<0.001

CD4^+^ (%)	Before	38.99 ± 1.65	Before	39.32 ± 1.68	1.086	0.280
	After	25.54 ± 1.68	After	30.55 ± 1.57	16.877	<0.001

CD4^+^/CD8^+^	Before	1.22 ± 0.35	Before	1.20 ± 0.31	0.331	0.741
	After	0.99 ± 0.01	After	1.87 ± 0.35	19.468	<0.001

**Table 3:** Comparison of patients' negative emotion scores ($\bar{\text{x}}$ ±*s*, points).

Group	SDS before after		SAS before after	
Intervention	59.64 ± 8.98	42.51 ± 8.57	60.11 ± 10.56	40.68 ± 6.98
Control	59.67 ± 8.87	48.65 ± 8.65	61.26 ± 10.57	47.65 ± 6.91
t	0.018	3.906	0.596	5.497
P	0.985	<0.001	0.552	<0.001

**Table 4:** Comparison of patient satisfaction with nursing [n(%)].

Group	Fully satisfied	Satisfied	Dissatisfied	Overall satisfaction
Intervention group	30 (50.0)	28 (46.7)	2 (3.3)	58 (96.7)
Control group	18 (30.0)	30 (50.0)	12 (20.0)	48 (80.0)
X^2^	5.000	0.134	8.086	8.086
P	0.025	0.715	0.004	0.004

## Data Availability

The data used to support the findings of this study are available on reasonable request from the corresponding author.
